The article "Aging Affects the Role of Myeloid-Derived Suppressor Cells in Alloimmunity" was published in 2022. Journal: Front Immunol.

# Aging Affects the Role of Myeloid-Derived Suppressor Cells in Alloimmunity

**DOI:** 10.3389/fimmu.2022.917972

**Published:** 2022-07-06

**Authors:** Andreas Schroeter, Maximilian J. Roesel, Tomohisa Matsunaga, Yao Xiao, Hao Zhou, Stefan G. Tullius

**Affiliations:** ^1^ Transplant Surgery Research Laboratory and Division of Transplant Surgery, Department of Surgery, Brigham and Women’s Hospital, Harvard Medical School, Boston, MA, United States; ^2^ Regenerative Medicine and Experimental Surgery, Department of General, Visceral and Transplant Surgery, Hannover Medical School, Hannover, Germany; ^3^ Institute of Medical Immunology, Charite Universitaetsmedizin Berlin, Berlin, Germany; ^4^ Department of Urology, Osaka Medical and Pharmaceutical University, Takatsuki City, Japan

**Keywords:** MDSC, myeloid cells, organ transplantation, alloimmunity, aging, immunosenescence

## Abstract

Myeloid-derived suppressor cells (MDSC) are defined as a group of myeloid cells with potent immunoregulatory functions that have been shown to be involved in a variety of immune-related diseases including infections, autoimmune disorders, and cancer. In organ transplantation, MDSC promote tolerance by modifying adaptive immune responses. With aging, however, substantial changes occur that affect immune functions and impact alloimmunity. Since the vast majority of transplant patients are elderly, age-specific modifications of MDSC are of relevance. Furthermore, understanding age-associated changes in MDSC may lead to improved therapeutic strategies. Here, we provide a comprehensive update on the effects of aging on MDSC and discuss potential consequences on alloimmunity.

## Introduction

Myeloid-derived suppressor cells (MDSC) are a heterogenous group of immature myeloid cells that exhibit immunosuppressive functions affecting various immune cells (1). First observed in patients with cancer, MDSC are generated under chronic pathological conditions including persistent inflammation or malignancies where continuous stimulation and inhibition of standard myelopoiesis pathways result in the formation of undifferentiated cells. Reflecting this heterogeneity, MDSC in mice are phenotyped as CD11b^+^Gr-1^+^ with two major subsets: granulocytic MDSC (G-MDSC) (CD11b^+^Gr-1^+^Ly6G^+^Ly6C^low^) and monocytic MDSC (M-MDSC) (CD11b^+^Gr-1^+^Ly6G^-^Ly6C^hi^), based on their expression of Ly6C and Ly6G (1–4). In humans, the classification is more complex with M-MDSC phenotyped as CD11b^+^CD33^+^CD14^+^CD66b^+^HLA-DR^low^ and G-MDSC as CD11b^+^CD33^+^CD14^-^CD15^+^HLA-DR^low^ cells (5). The functional capacities of these cells have gained increasing attention in the recent past. Most importantly, MDSC have shown a strong capacity to suppress CD4^+^ and CD8^+^ T-cell functions while promoting the activation and expansion of regulatory T cells (Tregs) (5–9). The mechanisms of immune modulation have also been shown to vary depending on the cell subset. Generally, G-MDSC suppress the immune function *via* reactive oxygen species (ROS) whereas the effects of M-MDSC are primarily mediated through the up-regulation of inducible nitric oxide synthase (iNOS), arginase, and immunosuppressive cytokines (10). However, immune modulation is not limited on the effects on T cells but also impacts innate immune cells including neutrophils, monocytes, macrophages, and dendritic cells (DCs) (11), many of which play a critical role in alloimmunity (12–16).

## Clinical Impact

In organ transplantation, MDSC may promote allograft acceptance and have therefore been of clinical interest in and beyond organ transplantation.

In various clinical settings including kidney, lung, and intestinal transplantation, significantly elevated levels of MDSC have been reported suppressing T-cell proliferation and pro-inflammatory cytokine levels when cultured *in vitro* (17–19). In addition, clinical studies investigating the role of MDSC in acute T-cell-mediated rejection (ATCMR) have shown an improved allograft function in parallel with increasing peripheral MDSC counts. In renal transplant biopsies, tissue injury has been attenuated with high peripheral MDSC counts, corroborating the immunosuppressive potential of MDSC in alloimmunity. Interestingly, MDSC collected from patients had the capacity to expand Tregs while inhibiting IL-17 production *in vitro* (20). Moreover, MDSC expansion correlated linearly with an increase in Tregs *in vivo* and Treg induction *in vitro* (21). Notably, transplant recipients with infections or chronic lung allograft dysfunction (CLAD) have shown lower G-MDSC levels when compared to patients with stable transplant function (18). Cytomegalovirus (CMV) infection, a major risk factor for developing CLAD, has been linked to an impaired MDSC differentiation (22, 23). In addition, hepatic stellate cells have been shown to induce MDSC both *in vivo* and *in vitro*, indicating the potential to promote liver allograft acceptance (24–27). Of additional interest, numbers of MDSC increased in intestinal transplant patients with acute cellular rejection (ACR) and positively correlated with serum IL-6 levels, a cytokine that has previously been shown to induce MDSC expansion (1). Furthermore, corresponding *in vitro* experiments have shown that IL-6 and methylprednisolone promoted the differentiation of bone marrow cells into MDSC. An accumulation of MDSC in the intestinal mucosa was also observed, and MDSC were able to suppress the T-cell-mediated destruction of donor intestinal epithelial organoids. Thus, MDSC may play an important role in suppressing the pathogenic T-cell response in the context of intestinal transplants and control ACR (19).

## Impact of Immunosuppressive Drugs on MDSC

In addition to the potential effects of MDSC on allograft survival, interactions with commonly used immunosuppressive drugs have been reported (**Table 1**). Clinically, circulating numbers of MDSC increased rapidly after applying calcineurin inhibitors, rapamycin, or corticosteroids (34, 35). Long-term, granulocytic subsets (G-MDSC) fluctuated in numbers whereas monocytic subsets (M-MDSC) remained relatively stable (38). Interestingly, M-MDSC from tacrolimus-treated but not from rapamycin-treated kidney transplant recipients were able to suppress the proliferation of CD4^+^ T cells, indicating that rapamycin may curtail the immunosuppressive abilities of M-MDSC (30). The correlation of MDSC activity with CNI levels may be explained by mechanistic findings that show an increased expression of indoleamine 2,3-dioxygenase (IDO), an enzyme regulating the immunosuppressive activity of MDSC, thereby inducing the suppressive functions of recipient MDSC (28). Conversely, rapamycin has been shown to downregulate IDO expression and may therefore also attenuate iNOS expression in rapamycin-exposed M-MDSC (30, 39).

**Table 1:** Effects of immunosuppressive drugs on MDSC in transplant models.

Class	Drug	Year	Model	Effects	Reference
CNI	CsA CsA Tacrolimus	2015 2016 2020	Kidney Tx Kidney Tx Kidney Tx	Immunosuppressive function ↑ Numbers ↑ / immunosuppressive function ↑ Numbers ↑ / immunosuppressive function ↑	[28] [29] [30]
mTORi	Rapa Rapa Rapa Rapa	2015 2017 2020 2021	Heart Tx Liver Tx Kidney Tx Skin Tx	Numbers ↑ / graft survival ↑ Numbers ↑ / immunosuppressive function ↑ Immunosuppressive function → Numbers ↑ / graft survival ↑ in obese recipients	[31] [32] [30] [33]
CS	Dex MP Dex Dex	2014 2018 2018 2018	Skin Tx ntestinal Tx Heart Tx Heart Tx	Numbers ↑ / immunosuppressive function ↑/ graft survival ↑ Differentiation ↑ / immunosuppressive function ↑ Numbers ↑ / graft survival ↑ / Tregs ↑ Immunosuppressive function ↑ Graft survival ↑ / Tregs ↑	[34] [19] [36] [37]

In other experiments, however, rapamycin has been shown to increase MDSC levels, enhancing cardiac and hepatic allograft survival in mouse models potentially facilitated through the induction of inducible iNOS (31, 32). Intriguingly, the adoptive transfer of MDSC from rapamycin-treated recipients prolonged allograft survival in third-party recipient mice (31). Most recently, delayed allograft rejection following MDSC induction by rapamycin has been shown in obese transplant recipients, emphasizing on the effectiveness of rapamycin in transplant recipients with preexisting conditions (33). As obesity has been linked to cellular senescence, those findings are of particular interest for the assessment of the role that MDSC may play in aging (40–42). Taken together, these findings may indicate that mTOR inhibition may have dual effects—both immunogenic as well as tolerogenic—on MDSC (30). Steroids have also been shown to impact MDSC numbers and functions (35). Steroid treatment correlates with increasing numbers of MDSC and Tregs in cardiac transplant models. Moreover, levels of Tregs were diminished when anti-Gr-1 antibodies targeting MDSC were administered in this study, emphasizing on the potential of MDSC affecting Tregs (36).

In addition, supplementing a granulocyte-macrophage colony-stimulating factor (GM-CSF) system with dexamethasone promoted MDSC with an enhanced immunosuppressive function specifically *in vitro*, and, when transferred into cardiac allograft recipients, prolonged allograft survival and Treg expansion. Mechanistically, iNOS and glucocorticoid receptor (GR) signaling pathways have been shown to be essential for mediating these processes. iNOS signaling was required for MDSC to regulate T-cell responses, whereas GR signaling was essential for mediating the recruitment of MDSC into allografts (37). The effects on MDSC were not only limited to rapamycin and corticosteroids as cyclosporine A also significantly increased the numbers and immunosuppressive functions of MDSC, ameliorating alloimmune responses (29).

## MDSC in Alloimmunity

Organ tpransplantation initiates a complex immunological cascade composed of cellular and humoral components, ultimately leading, if not successfully treated or modified, to an irreversible rejection. In addition to the adaptive immune system, several components of the innate immune response including dendritic cells (DCs), natural killer (NK) cells, and macrophages play critical roles in this process (43, 44). Accumulating evidence suggests that MDSC may also play an important role in allorecognition. Experimental models including kidney, heart, and skin transplantation have shown elevated numbers of MDSC that can suppress T-cell proliferation while inducing apoptosis, linked to graft prolongation (39, 45–47). It has been demonstrated that MDSC are recruited from the bone marrow, migrating into the graft early after transplantation (47). Interestingly, graft survival was prolonged in old mice and those exhibiting high serum levels of TGF-β, an immunosuppressive cytokine that has been shown to increase with age (39, 46).. When entinostat, a histone deacetylase inhibitor, was administered to block MDSC function, graft survival was abbreviated comparable to survival times observed in young mice (48). In a pre-sensitized transplant model, massively elevated levels of MDSC were found in the peripheral blood of recipient mice. Notably, particularly the CD11b^+^Gr-1^(-low)^ subtype has been shown to prevent allograft injury after prolonged ischemia (49). *In vitro* experiments have shown that these effects are dependent on iNOS, an enzyme that is upregulated in graft-infiltrating MDSC (16, 45). Additional supporting evidence comes from findings showing that the suppressive ability of MDSC is mediated by nitric oxide (NO), secreted subsequent to receiving signals from activated T cells including IFN-γ and contact-dependent stimuli (16). Additional experiments in iNOS knockout mice demonstrated that the inhibition of activated T cells in lymphoid organs depended on NO (50). In support of clinical findings, MDSC play also a critical role in initiating the beneficial effects of Tregs with CCL5 secreted by graft infiltrating MDSC promoting the accumulation of Tregs in tolerant kidney allografts (20, 21, 51). Conversely, boosting Tregs increased the numbers of CD11b^+^Gr-1^(-low)^ MDSC in recipient peripheral blood, spleen, and the graft itself (49).

Adoptive transfer experiments demonstrated that the expansion of MDSC is initiated by the inhibitory receptor immunoglobulin-like transcript (ILT)-2 and its ligands leading to prolonged allograft survival (52). Other cytokines including IL-2C, IL-33, and TNF-α have also been shown to induce MDSC resulting in a suppression of T-cell activation (53–56). Additional studies confirmed these findings; however, no alterations of antigen-specific CD8^+^ T-cell proliferation and cytotoxicity were found (57, 58). Based on previous findings, the combinatorial application of induced MDSC and Tregs exhibited superior immunosuppressive capabilities with prolonged graft survival compared to the treatment with individual cell populations (53). Notably, other regulatory myeloid cell types including tolerogenic dendritic cells and regulatory/suppressor macrophages have also been shown to prolong skin allograft survival by distinct mechanisms of action (59).

## The Role of MDSC in Ischemia–Reperfusion Injury

Ischemia–reperfusion injury (IRI) is an inevitable component of solid organ transplantation. In general, pro-inflammatory events are initiated upon blood flow cessation and resumption causing a myriad of immune cells to migrate into the graft. As an immediate response, innate immune cells including neutrophils and macrophages infiltrate the organ, secreting pro-inflammatory cytokines while initiating phagocytosis and complement activation (60–62). Adaptive immune cells such as T and B cells contribute to the deleterious events by producing pro-inflammatory cytokines, lysosomal enzymes, and ROS (63–65). Recent data indicate that MDSC may also play an important role in IRI. In murine kidney transplant models, MDSC have been found to aggravate IRI. These findings may be explained by the differentiation of M-MDSC into harmful macrophages and dendritic cells (66). However, the immunosuppressive effects that MDSC exert on adaptive CD4^+^ and CD8^+^ T cells were not sufficient to prevent an impairment of renal function. Supporting evidence comes from findings that pharmacological depletion of MDSC in kidney IRI models using anti-Gr-1 antibodies entailed beneficial effects. Interestingly, human C-reactive protein (CRP), which has previously been found to exacerbate renal IRI, has been shown to specifically promote the kidney infiltration of G-MDSC, a subtype displaying augmented immunosuppressive activities. Consistently, blocking CRP reduced the numbers of G-MDSC and attenuated albuminuria, suggesting a regulating role of CRP in MDSC activation (67). In contrast, increased renal infiltration of MDSC upon granulocyte colony-stimulating factor (G-CSF) administration improved renal function after IRI and attenuated acute tissue injury as well as chronic renal fibrosis (68, 69). In addition, further mechanistic studies have shown that renal fibrosis can be alleviated by MDSC through CCL5-CCR-5 axis regulation and TGF-β1/Smad/Snail signaling pathway inhibition (70).

## Changes of MDSC in Aging

Aging is characterized by an increased accumulation of proinflammatory cytokines together with modifications of the composition and the effects of various immune cell types of both the adaptive and innate immune systems (71, 72). In general, adaptive immune function appears modified in aging, manifesting clinically with a compromised response to vaccines and a limited capacity to combat infections (73). At a cellular level, thymic involution leads to a decreased production of naïve T cells in the elderly with a restricted T-cell receptor repertoire. In addition, functional impairments of naïve CD4 T cells that include a compromised proliferation upon stimulation by antigen-presenting cells in addition to a limited cytokine production have been observed. Consistently, effector functions have been inferior when compared to cells derived from young progenitors (74). In parallel, B-cell production also declines with age and an accumulation of phenotypically distinct, age-associated B cells has been reported (75–77). These findings are in line with functional limitations, leading to an impaired capacity to mount sufficient antibody responses (78). Furthermore, functional changes in natural killer T cells (NKT cells) have been observed in elderly individuals (79). In addition to changes in the adaptive immune response, alterations of innate immune cells have also been found. Macrophages from old mice have shown a reduced production of pro-inflammatory cytokines following stimulation by lipopolysaccharides (LPS) (80–83). These findings may be attributed to various age-related changes including a reduced Toll-like receptor (TLR) expression, decreased nuclear factor kappa B (NF-κB) and mitogen-activated protein kinase (MAPK) activation, and increased levels of the signaling protein A20, which blocks TRAF6 signaling, thus interfering with the TLR4 pathway (82, 84–88). In addition, an impaired cytokine production by DCs and monocytes upon stimulation has been reported (89, 90). MDSC are considered progenitors of innate immune cells and increase in numbers with aging (**Figure 1**) (91, 92). Elevated numbers of MDSC have been shown to accumulate in the blood, bone marrow, and secondary lymphoid organs in aging and may, in fact, through the initiation of a defective PI3K-Akt signaling pathway contribute themselves to immune senescence (93, 94). Further experimental studies suggest that the expansion of MDSC with aging relies, at least in part, on NF-κB activation (95). In addition, a shift toward myelopoiesis in bone marrow hematopoietic stem cells (HSC) occurs with aging and may further promote the increase of MDSC in elderly individuals (96). Moreover, MDSC could increase myelopoiesis themselves by secreting TGF-β, a cytokine which promotes the differentiation of hematopoietic stem cells into myeloid cells (97). Consistently, elevated numbers of MDSC have also been shown in older humans with elevated levels of proinflammatory cytokines including TNF-α, IL-6, and IL-1β necessary for MDSC differentiation. Interestingly, elderly individuals with a history of cancer showed significantly higher levels of MDSC in the peripheral blood, pointing toward a role of MDSC in cancer development (6–8, 98). Additional evidence comes from clinical studies that also observed elevated numbers of MDSC with a predominance of the granulocytic subtype in old individuals (99). At a functional level, older MDSC isolated from spleen and bone marrow have shown an augmented ability to inhibit T-cell functions when compared with MDSC from young donors. Consistently, removal of MDSC from aged splenocyte cultures restored T-cell proliferation *in vitro* and was associated with reduced NO levels (93). Additional supporting evidence comes from studies showing a correlation between increased MDSC levels in old mice and limited T-cell tumor cytotoxicity. In addition, MDSC also delayed the response to tumor cells when adoptively transferred to young mice. Mechanistically, age-associated induction of arginase 1 in MDSC may play an important role in suppressing T-cell functions (100). Thus, age-related changes in MDSC and their subsequent impact on other immune cells may influence allograft tolerance in various ways. In addition, age-associated limited Th1 alloimmunity may enhance the effects by older MDSC (101). Moreover, suppressive capacities of Tregs have been found to be well-preserved experimentally, thus promoting graft acceptance (101). At a molecular level, an augmented expression of senescent cell markers p16 and p21 has been found in aging MDSC. However, other senescence-associated phenotypes including the accumulation of γH2AX and 53BP1 foci, reduced lamin B1 expression, and induced IL-6 expression have not been detected. Moreover, senolytics (ABT-263) were unable to eliminate these cells (102).

**Figure 1:** Aging affects the role of MDSC in alloimmunity. Changes in MDSC numbers and functionality occur during aging. Environmental factors including elevated cytokine levels, increased myelopoiesis, and malignancies impact MDSC numbers. Those effects impact alloimmunity in multiple ways including T-cell suppression, Treg activation and migration, and aggravating IRI.

Overall, senescence of MDSC remains ill-defined currently. Age-related changes in MDSC favoring a generally immunosuppressive environment may have beneficial effects in transplantation, ameliorating alloimmunity in older recipients.

## Therapeutic Strategies

Over the recent past, therapeutic strategies utilizing MDSC have been proposed for various immune-related diseases (103). In cancer, MDSC contribute to tumor progression, metastasis development, and resistance to immunotherapeutic drugs by establishing an immunosuppressive microenvironment (104, 105). Thus, various therapeutic strategies including the depletion of MDSC, blocking MDSC migration, and attenuating their immunosuppressive capacities have been tested (106–109). Autoimmune diseases such as multiple sclerosis, myasthenia gravis, and rheumatoid arthritis have also been shown to be associated with changes in MDSC, and corresponding therapeutic strategies have been proposed (110–113). In transplantation, adoptive transfer of MDSC has yielded promising results in various experimental models (56, 114, 115). Promoting the accumulation of MDSC through nanoimmunotherapy targeting myeloid cell precursors demonstrated graft tolerance in most recipient animals. Intriguingly, the effect was already present after short-term administration of the nanobiologics (116). Further supporting evidence comes from other experimental models in which adoptively transferred MDSC were found to expand after transplantation, migrating into the graft and prolonging allograft survival (117). Moreover, MDSC facilitated the recruitment of Tregs into cardiac allografts by inducing programmed death ligand-1 (PD-L1) (118). It needs to be stressed, however, that not all studies confirmed the effects of MDSC on graft prolongation (45, 119). MDSC have thus far not been tested clinically in transplant patients. Notably, MDSC may lose their immunosuppressive functions in an already immune-activated environment as MDSC transferred into patients with acute graft-versus-host-disease lost their suppressive capacity and their potential to improve transplant outcomes. Mechanistically, an inflammasome-induced differentiation of MDSC into mature cells may play a role (120). In addition to bone marrow-derived MDSC, induced pluripotent stem cells (iPSC) have been evaluated for their immunosuppressive potential. Interestingly, fibroblast-derived iPSC cultured in medium containing GM-CSF, M-CSF, IL-4, and LPS have been able to suppress allogeneic T- as well as B-cell response while reducing alloantibody production *in vivo* (111, 121).

Taken together, MDSC cell therapy may, at least in theory, have immunosuppressive potential in organ transplantation; however, confirmatory clinical studies are missing (58).

## Conclusion

MDSC have a profound impact on immune responses. While the immunosuppressive capacities of MDSC may have potential in clinical transplantation, effects need to be confirmed. Side effects including an increased risk for malignancies need to be carefully assessed (122). Aging impacts both MDSC numbers and functionality with potential consequences on their capacity to modulate immune responses. Understanding those aspects in greater detail may contribute to novel therapeutic strategies for improving allograft survival in an age-specific fashion (45, 56, 58, 123, 124). Moreover, monitoring the frequencies of MDSC as biomarkers in organ transplant recipients may provide additional valuable diagnostic information.

## Author Contributions

All authors listed have made a substantial, direct, and intellectual contribution to the work, and approved it for publication.

## Funding

This work was supported by the Biomedical Education Program BMEP (to AS and MJR), NIH grants R01AG064165 and U01AI132898 (to SGT) and P30AG031679 (to HZ).

## Conflict of Interest

The authors declare that the research was conducted in the absence of any commercial or financial relationships that could be construed as a potential conflict of interest.

## Publisher’s Note

All claims expressed in this article are solely those of the authors and do not necessarily represent those of their affiliated organizations, or those of the publisher, the editors and the reviewers. Any product that may be evaluated in this article, or claim that may be made by its manufacturer, is not guaranteed or endorsed by the publisher.
